This article has been retracted.

# The effects of intermittent bolus paravertebral block on analgesia and recovery in open hepatectomy: a randomized, double-blinded, controlled study

**DOI:** 10.1186/s12893-023-02125-0

**Published:** 2023-08-05

**Authors:** Jin Wang, Xulei Cui, Yuelun Zhang, Xinting Sang, Le Shen

**Affiliations:** 1 Department of Anesthesiology, Peking Union Medical College Hospital, Chinese Academy of Medical Sciences, Beijing, China; 2 Center Research Lab, Peking Union Medical College Hospital, Chinese Academy of Medical Sciences, Beijing, China; 3 Department of Hepatology, Peking Union Medical College Hospital, Chinese Academy of Medical Sciences, Beijing, China; 4 State Key Laboratory of Complex Severe and Rare Disease, Beijing, China

**Keywords:** Nerve block, Hepatectomy, Pain, Postoperative, Enhanced recovery after surgery, Analgesia, Patient-controlled, Acute pain, Chronic pain, Anesthesia

## Abstract

**Background:**

We aimed to investigate the effects of intermittent bolus paravertebral block on analgesia and recovery in open hepatectomy.

**Methods:**

Eighty 18–70 years old, American Society of Anesthesiologists level I-III patients scheduled for hepatectomy with a J-shaped subcostal incision were enrolled and randomized to receive either intermittent bolus paravertebral ropivacaine (0.5% loading, 0.2% infusion) or 0.9% saline infusion at 1:1 ratio (25 ml loading before surgery, 0.125 ml/kg/h bolus for postoperative 48 h). The primary outcome was set as postoperative 48 h cumulative intravenous morphine consumption recorded by a patient-controlled analgesic pump.

**Results:**

Thirty-eight patients in each group completed the study. The cumulative morphine consumptions were lower in the paravertebral block than control group at postoperative 24 (difference -10.5 mg, 95%CI -16 mg to -6 mg, *P* < 0.001) and 48 (difference -12 mg, 95%CI -19.5 mg to -5 mg, *P* = 0.001) hours. The pain numerical rating scales at rest were lower in the paravertebral block than control group at postoperative 4 h (difference -2, 95%CI -3 to -1, *P* < 0.001). The active pain numerical rating scales were lower in the paravertebral block than control group at postoperative 12 h (difference -1, 95%CI -2 to 0, *P* = 0.005). Three months postoperatively, the paravertebral block group had lower rates of hypoesthesia (OR 0.28, 95%CI 0.11 to 0.75, *P* = 0.009) and numbness (OR 0.26, 95%CI 0.07 to 0.88, *P* = 0.024) than the control group.

**Conclusions:**

Intermittent bolus paravertebral block provided an opioid-sparing effect and enhanced recovery both in hospital and after discharge in patients undergoing hepatectomy.

**Trial registration:**

clinicaltrials.gov (NCT04304274), date: 11/03/2020.

## Background

Paravertebral block has been used as an effective perioperative analgesic approach in many types of surgeries, such as thoracic, breast, cardiac and abdominal surgeries [1–5]. It has an opioid-sparing effect and provides good pain relief. Compared to epidural analgesia, paravertebral block carries a lower risk of multiple complications, including hypotension, nausea, vomiting, pruritus and urinary retention [2, 6].

Open hepatectomy often causes severe pain due to its large incision and extensive surgical damage. Cases of paravertebral block use in hepatectomy have been reported [7, 8], but clinical studies were limited [9, 10]. Furthermore, the effect of paravertebral block on persistent post-surgical pain remains controversial [11, 12]. To the best of our knowledge, the current literature does not include any study reporting the effects of intermittent bolus paravertebral block on intraoperative management, postoperative analgesia and recovery both in hospital and after discharge in patients undergoing open hepatectomy.

This study aimed to investigate the effects of intermittent bolus paravertebral block on analgesia and recovery in patients undergoing open hepatectomy for hepatic tumors. We hypothesized that intermittent bolus paravertebral block reduced postoperative 48 h cumulative intravenous opioid consumption. Intraoperative management, postoperative analgesia and recovery, and follow-up data were collected and compared between patients with and without paravertebral block. We present the following article in accordance with the CONSORT reporting checklist.

## Methods

### Study design

This is a prospective, randomized, controlled, double-blinded study. The study design was approved by the hospital’s institutional review board (ZS-1031) and registered at Clinicaltrial.gov (NCT04304274, date 11/03/2020).

### Participants and settings

The study was conducted in a tertiary hospital in Beijing, China. Patients undergoing open hepatectomy for hepatic tumors were screened for eligibility. Inclusion criteria were: (1) 18–70 years old; (2) American Society of Anesthesiologists physical status I-III; (3) hepatectomy with a J-shaped subcostal incision; (4) informed consent signed. Exclusion criteria were: (1) allergic to medications used; (2) coagulopathy or on anticoagulants; (3) recent or long-term use of analgesics; (4) participating in other trials or unable to cooperate.

### Randomization, allocation and blinding

Patients were randomly assigned to paravertebral block or control group at a 1:1 ratio based on the results of a computerized randomization program generated by a statistician. The allocation results were sealed in opaque envelopes and stored in the research center. Analgesic pumps with either ropivacaine or saline were prepared by nurses uninvolved in any other part of the study. The patients, surgeons, anesthesiologists and postoperative follow-up assessors were blinded to the group assignments. Unmasking was performed after the completion of statistical analysis.

### Interventions

Patients’ baseline characteristics were evaluated during preoperative visits. The anesthesiologists educated the patients on the anesthetic process, use of analgesic pumps, 0 to10 points pain numerical rating scale (NRS) with 0-point indicating no pain and 10-point indicating the maximum degree of insufferable pain, and collected the patients’ preoperative pain NRS of the surgical sites.

Thoracic paravertebral space catheterization was performed 30 min before anesthesia (Fig. 1). The patient was placed in a lateral position with peripheral venous access. After sterilization, an in-plane approach [13] was used to insert a 21-gauge 10 cm needle (PlexoLongNanoline; Pajunk Inc, Geisingen, Germany) into the T8 paravertebral space between the internal intercostal membrane and the pleura under the guidance of ultrasonography (X-port, Sonosite Inc., USA). After a negative aspiration test, 25 ml of transparent study solution was injected into the paravertebral space. Then, a catheter (PlexoLongNanoline; Pajunk Inc, Geisingen, Germany) was inserted through the needle into the paravertebral space, secured with Bio-gel to the patient’s back. The catheter was connected to a programmable, portable, electronic infusion pump (Apon ambulatory infusion pump ZZB-I, Jiangsu Apon Medical Technology Co., Ltd.) to deliver a bolus of 0.125 ml/kg transparent study solution per hour over 90 s, commencing immediately after surgery.

**Fig. 1:** Ultrasound-guided paravertebral block. P: Pleura, L: Lamina, *: Local anesthetics.

Paravertebral block group patients used 25 ml of 0.5% ropivacaine as initial loading dose and continued with 0.2% ropivacaine as subsequent intermittent bolus dose. Control group patients used 25 ml 0.9% saline as initial loading dose and continued with 0.9% saline as subsequent intermittent bolus dose. To avoid inadvertent unmasking of the allocation, the extent of sensory block was not tested.

After paravertebral block, general anesthesia with endotracheal intubation was performed with intravenous fentanyl (2 μg/kg), propofol (1.5–2.0 mg/kg) and rocuronium (0.6 mg/kg). Anesthesia was maintained with sevoflurane and a 50%O_2_-50%N_2_O mixture to maintain a BIS index within 40 to 60. Atracurium was infused to maintain muscle relaxation and ceased 30 min before the end of surgery. Fentanyl was given in 1 μg/kg per bolus to maintain heart rate and blood pressure below 120% of its preoperative levels. The same surgical team used the “CUSA” technique to perform standard hepatectomy with a J-shaped right subcostal incision. The J-shaped incision consisted of a right subcostal incision with a medial cranial extension to the xiphoid process and a right lateral extension with transection of the oblique abdominal musculature [14]. Upon completion of the surgery, sevoflurane and N_2_O were discontinued and the neuromuscular blockade was reversed with neostigmine (50 μg/kg). Extubation was carried out when the patient was fully awake.

Patient-controlled intravenous morphine pump (Gemstar, Hospiria Inc., USA) was connected to the patient after extubation. Intravenous morphine was given with no background infusion, 1–2 mg per bolus, 5-min lockout interval and an upper limit of 8 mg per hour. If the patient still complained about pain with the upper limit dose, an intravenous Cox-2 inhibitor was given as rescue analgesia. Both paravertebral and intravenous analgesia was provided until 48 h postoperatively. All patients received same postoperative recovery program including daily crystalloid and nutrition infusion, oral clear fluid intake on postoperative day one and food intake after passing gas. No laxatives were given before oral food intake. If catheter dislocation happened, re-catheterization was decided by the patient. Two trained clinicians visited the patients and assessed the outcomes in the ward at postoperative 2, 4, 12, 24 and 48 h. Follow-up after discharge was completed via clinical visits or telephones at postoperative 3 months.

### Outcomes and definitions

The primary outcome was set as cumulative morphine consumption at postoperative 48 h and collected from analgesic pump records. Secondary outcomes included: (1) postoperative 2-, 4-, 12- and 24-h cumulative morphine consumptions; (2) postoperative 0-, 2-, 4-, 12-, 24- and 48-h rest and active pain NRS; (3) opioid-related adverse effects such as respiratory depression, pruritus, nausea, vomiting, urinary retention recorded as Foley catheter removal time and bowel movement recorded as gas time; (4) postoperative 48-h recovery status including cold feeling, thirst, drowsiness, shiver and cognitive decline. The recovery parameters were evaluated with a 0–3 points Likert scale with 0-point defined as none, 1-point defined as mild, 2-point defined as moderate and 3-point defined as severe. Overall, analgesia and emergence satisfaction were evaluated with a 1–5 points Likert scale with 1-point defined as very unsatisfied and 5-point defined as very satisfied; (5) Postoperative three months recovery status including rates of pain, numbness and hypoesthesia at the surgical site, sleep disorder, rest and active pain NRS, and pain characteristics.

### Sample size and statistical analysis

The study sample size was calculated based on the result of a pilot study. The mean postoperative 48 h cumulative morphine consumptions were (16.8 ± 13.5) mg in the paravertebral block group and (32.7 ± 19.2) mg in the control group. Thirty-five patients were required in each group to achieve an α level of 0.01 and β level of 0.9. Considering possible dropouts, a total of 80 patients were enrolled.

Statistical analysis was performed using SPSS for Mac version 23.0 (IBM Corp., Armonk, NY, USA). Normality was tested using the Q-Q plots. Normally distributed variables were expressed as mean ± SD, non-normally distributed variables were expressed as median (quartile), and categorical variables were expressed as frequency (percentage). Normally distributed continuous data were analyzed using the independent *t-test* and non-normally distributed continuous data were analyzed using the Mann–Whitney U tests. Categorical data were compared using the *Chi*-square test when the expected cell counts > 5, otherwise, the *Fisher’s e*xact test was used. All tests were two-tailed, and a *P* value less than 0.05 was considered statistically significant.

## Results

From Mar 2020 to Dec 2021, a total of ninety-four patients were screened and eighty were eligible for the study. Nine patients did not meet the inclusion criteria due to advanced age, coagulation dysfunction and language barrier. Five patients refused to participate in the study. After allocation, two patients in the control group failed the intervention due to change of surgical plan. All patients in the paravertebral block group successfully received study intervention. During follow-up, two patients in the paravertebral block group were dropped due to catheter dislocation and unplanned ICU admission. No nerve block-related adverse events occurred. All patients in the control group completed the follow-up. Finally, thirty-eight patients in each group were entered into analysis (Fig. 2).

**Fig. 2:** Consolidated standards of reporting trials flow diagram showing patient progress through the study phases.

### Baseline data

Baseline clinical characteristics were listed in Table 1. The age, sex, body mass index, ASA classification, preoperative pain score, neuropathy and severe sleep disorder history, hemoglobin and platelet counts, liver function and coagulation test results were similar between the paravertebral block and control groups (all* P* > 0.05).

**Table 1:** Baseline characteristics of the paravertebral block and control groups

	PVB group (*n* = 38)	Control group (*n* = 38)
Age (years)	55 ± 11	56 ± 10
Male (n, %)	22, 57.9%	23, 60.5%
BMI (kg•m^−2^)	23.31 ± 3.15	23.60 ± 3.63
ASA I/II/III level	19/18/1	15/22/1
Pain NRS	0 (0,1)	0 (0, 0)
Neuropathy	0, 0.0%	0, 0.0%
Severe sleep disorder	0, 0.0%	0, 0.0%
Hemoglobin (g•L^−1^)	139 ± 19	141 ± 19
Platelet (× 10^9^•L^−1^)	203 ± 87	179 ± 69
ALT (U•L^−1^)	31 ± 24	31 ± 25
Albumin (g•L^−1^)	42 ± 6	43 ± 4
Creatinine (μmol•L^−1^)	72 ± 16	72 ± 14
PT (s)	13 ± 1	12 ± 1
APTT (s)	29 ± 4	28 ± 5

*PVB* Paravertebral block, *BMI* Body mass index, *ASA* American Society of Anesthesiologists, *NRS* Numerical rating scale (0–10 points), *ALT* Alanine aminotransferase, *PT* Prothrombin time, *APTT* Activated prothrombin time

### Intraoperative data

Intraoperative data were listed in Table 2. The baseline heart rate and blood pressure were defined as the average values of it measured by 3 alternative times preoperatively in ward. In the paravertebral block group, the intraoperative arterial pressure and heart rate were similar to its baseline levels (*P* > 0.05). In the control group, the intraoperative arterial blood pressure was similar to its baseline level(*P* > 0.05), but the intraoperative heart rate was lower (difference 4 bpm, 95%CI 2 to 7 bpm, *P* = 0.003) than its baseline level.

**Table 2:** Operation data of the paravertebral block and control groups

	PVB group (*n* = 38)	Control group (*n* = 38)	Difference 95% CI	*P* value
Surgical time (hours)	2.9 ± 0.9	3.0 ± 1.1	-0.2 (-0.6, 0.3)	0.518
Baseline HR (bpm)	77 ± 9	76 ± 8	2 (-2, 5)	0.393
Baseline MAP (mmHg)	91 ± 8	93 ± 9	-2 (-6, 2)	0.350
Mean HR (bpm)	76 ± 11	71 ± 10	5 (0, 9)	0.053
Mean MBP (mmHg)	89 ± 8	93 ± 9	-4 (-8, 0)	0.031*
Mean Sevoflurane (MAC)	1.1 ± 0.2	1.2 ± 0.2	-0.1 (-0.2, 0.0)	0.020*
Awake time (min)	8 ± 5	8 ± 5	0 (-2, 2)	0.961
Extubation time (min)	12 ± 6	10 ± 6	2 (-1, 4)	0.181
Fentanyl (μg)	332 ± 107	371 ± 125	-40 (-93, 13)	0.140
Ephedrine (mg)	6 (6, 16)	6 (0, 7)	6 (0,6)	0.004*
Phenylephrine (ug)	0 (0, 25)	0 (0, 0)	0 (0,0)	0.255
Urapidil (mg)	0 (0, 0)	0 (0, 0)	0 (0,0)	0.301
Atropine (mg)	0 (0, 0)	0 (0, 0)	0 (0,0)	0.089
Crystalloid (ml)	1800 (1525, 2300)	1800 (1300, 1925)	400 (0, 500)	0.024*
Colloid (ml)	0 (0, 500)	500 (0, 500)	0 (0,0)	0.595
RBC (U)	0 (0, 0)	0 (0, 1)	0 (0,0)	0.781
Plasma (ml)	0 (0, 0)	0 (0, 0)	0 (0,0)	0.838
Urine (ml)	675 (375, 1125)	350 (200, 600)	300 (100, 500)	0.002*
Hemorrhage (ml)	275 (100, 400)	200 (139, 425)	0 (-100, 100)	0.805

*PVB* Paravertebral block, *D* Difference, *CI* Confidential interval, *HR* Heart rate, *MBP* Mean blood pressure, *RBC* Red blood cell

^*^Significant statistical difference

As for between-group comparison, paravertebral block group had lower arterial blood pressure (difference -4 mmHg, 95%CI -8 to 0 mmHg, *P* = 0.031), used less sevoflurane (difference -0.1MAC, 95%CI -0.2MAC to 0.0MAC, *P* = 0.020) but more ephedrine (difference 6 mg, 95%CI 0 to 6 mg, *P* = 0.004) than control group. However, the 0.1MAC between-group difference in sevoflurane consumption was considered of no clinical significance. Other medications used were similar between the two groups (all *P* > 0.05). Paravertebral block group infused larger volume of crystalloid (difference 400 ml, 95%CI 0 to 500 ml, *P* = 0.024) than control group, but its urine output volume (difference 300 ml, 95%CI 100 ml to 500 ml, *P* = 0.002) was also higher than that of control group. The volumes of colloid infusion, blood products transfusion and hemorrhage were similar between the two groups (all *P* > 0.05).

### Postoperative data

Postoperative analgesia data were listed in Table 3 and depicted in Fig. 3. The cumulative morphine consumptions at postoperative 2 (difference -2.5 mg, 95%CI -3.5 mg to -1.5 mg, *P* < 0.001), 4 (difference -3.5 mg, 95%CI -4.5 mg to -1.5 mg, *P* < 0.001), 12 (difference -6.5 mg, 95%CI -10 mg to -3.5 mg, *P* < 0.001), 24 (difference -10.5 mg, 95%CI -16 mg to -6 mg, *P* < 0.001) and 48 (difference -12 mg, 95%CI -19.5 mg to -5 mg, *P* = 0.001) hours were lower in the paravertebral block than control group. Rescue analgesia rate was also lower in the paravertebral block than control group (OR 0.29, 95%CI 0.08 to 1.00, *P* = 0.044).

**Table 3:** Postoperative cumulative morphine consumption and pain NRS score at rest and on movement of the paravertebral block and control group at different time points

Time points	PVB group (*n* = 38)	Control group (*n* = 38)	Difference 95%CI	*P* value
Morphine (mg)				
2 h	1.5 (1.0, 2.3)	4.5 (1.5, 6.0)	-2.5 (-3.5, -1.5)	< 0.001*
4 h	1.5 (1.5, 4.5)	6.0 (3.0, 9.1)	-3.5 (-4.5, -1.5)	< 0.001*
12 h	5.0 (1.5, 12.0)	12.5 (7.1, 21.3)	-6.5 (-10, -3.5)	< 0.001*
24 h	10.0 (4.5, 18.0)	19.8 (13.1, 33.4)	-10.5 (-16, -6)	< 0.001*
48 h	15.8 (5.6, 28.5)	26.5 (17.8, 45.6)	-12 (-19.5, -5)	0.001*
Rest NRS				
0 h	0 (0, 0)	3 (0, 5)	-2 (-3,-2)	< 0.001*
2 h	2 (0, 3)	3 (3, 5)	-2 (-3,-1)	< 0.001*
4 h	2 (0, 3)	3 (2, 4)	-2 (-3,-1)	< 0.001*
12 h	2 (2, 3)	3 (2, 3)	0 (-1,0)	0.229
24 h	2 (1, 3)	2 (2, 3)	0 (-1,0)	0.352
48 h	1 (0, 2)	1 (0,2)	0 (-1,0)	0.495
Active NRS				
0 h	0 (0, 1)	4 (3, 6)	-3 (-4,-2)	< 0.001*
2 h	3 (1, 4)	4 (3, 6)	-2 (-3,-1)	0.001*
4 h	3 (1, 4)	4 (3, 5)	-1 (-2,-1)	< 0.001*
12 h	3 (2, 4)	4 (3, 5)	-1 (-2,0)	0.005*
24 h	4 (2, 5)	4 (3, 5)	0 (-1,1)	0.650
48 h	2 (2, 3)	3 (2, 4)	-1 (-1,0)	0.081

*PVB* Paravertebral block, *h* hours, *NRS* Numerical rating scale

^*^Significant statistical difference

**Fig. 3:** **a** Postoperative morphine consumption at different time points. **b** Postoperative pain numerical rating scale at rest at different time points. **c** Postoperative active pain numerical rating scale at different time points.

The pain NRS scores at rest were lower in the paravertebral block than control group at postoperative 0 (difference -2, 95%CI -3 to -2, *P* < 0.001), 2 (difference -2, 95%CI -3 to -1, *P* < 0.001) and 4 (difference -2, 95%CI -3 to -1, *P* < 0.001) hours, and similar between the two groups at postoperative 12, 24 and 48 h (all *P* > 0.05). The active pain NRS scores were lower in the paravertebral block than control group at postoperative 0 (difference -3, 95%CI -4 to -2, *P* < 0.001), 2 (difference -2, 95%CI -3 to -1, *P* = 0.001), 4 (difference -1, 95%CI -2 to -1, *P* < 0.001) and 12 (difference -1, 95%CI -2 to 0, *P* = 0.005) hours, but similar between the two groups at postoperative 24 and 48 h (*P* > 0.05).

Postoperative recovery data during hospital stay and three months after discharge were listed in Table 4 and 5. At postoperative 48-h, paravertebral block group had lower drowsiness score (difference 0, 95%CI -1 to 0, *P* = 0.006) and higher emergence satisfaction score (difference 0, 95%CI 0 to 1, *P* = 0.019) than control group. Other recovery data including nausea, vomiting, pruritus, respiratory depression, bowel movement, Foley catheter removal, thirst, cold feeling, cognitive decline, shivering, analgesia and overall satisfaction, and the length of hospital stay were similar between the two groups (all *P* > 0.05).

**Table 4:** In-hospital recovery data of the paravertebral block and control group

	PVB group (*n* = 38)	Control group (*n* = 38)	OR / Difference 95% CI	*P* value
Rescue analgesia (n, %)	4, 10.5%	11, 28.9%	0.29 (0.08, 1.00)	0.044*
Nausea (n, %)	23, 60.5%	18, 47.4%	1.70 (0.69, 4.23)	0.250
Vomiting (n, %)	4, 10.5%	8, 21.0%	2.27 (0.62, 8.29)	0.208
Pruritus (n, %)	3, 7.9%	3, 7.9%	1.00 (0.19, 5.30)	1.000
Respiratory depression (n, %)	7, 18.4%	14, 36.8%	0.39 (0.14, 1.11)	0.073
Bowel movement (hours)	60 ± 28	60 ± 21	0 (-11, 11)	0.979
Foley catheter removal (hours)	40 ± 23	46 ± 23	-5 (-16, 5)	0.270
Drowsiness (points)	0 (0, 1)	1 (0, 1)	0 (-1,0)	0.006*
Thirsty (points)	1 (1, 2)	1 (1, 2)	0 (-1, 0)	0.883
Feel cold (points)	0 (0, 0)	0 (0, 0)	0 (0, 0)	0.267
Cognitive decline (points)	0 (0, 0)	0 (0, 0)	0 (0, 0)	0.330
Shiver (points)	0 (0, 0)	0 (0, 0)	0 (0, 0)	0.969
Emergence satisfaction (points)	5 (4, 5)	4 (4, 5)	0 (0,1)	0.019*
Analgesia satisfaction (points)	4 (4, 5)	4 (4, 5)	0 (0, 0)	0.200
Overall satisfaction (points)	5 (4, 5)	4 (4, 5)	0 (0, 0)	0.262
Hospital stay(days)	9 ± 5	10 ± 4	-1 (-3, 1)	0.202

*PVB* Paravertebral block, *OR* Odds ratio, *D* Difference, *CI* Confidential interval

^*^Significant statistical difference

**Table 5:** Postoperative three months recovery data of the paravertebral block and control group

	PVB group (*n* = 38)	Control group (*n* = 38)	OR 95% CI	*P* value
Hypoesthesia (n, %)	9, 23.7%	20, 52.6%	0.28 (0.11, 0.75)	0.009*
Numbness (n, %)	4, 10.5%	12, 31.6%	0.26 (0.07, 0.88)	0.024*
Pain (n, %)	18, 47.4%	15, 39.5%	1.38 (0.56, 3.43)	0.488
Rest pain NRS (points)	0 (0, 3)	0 (0,0)	0 (0,0)	0.147
Active pain NRS (points)	0 (0, 3)	1 (0, 3)	0 (-3, 0)	0.762
Throbbing pain (n, %)	3, 7.9%	1, 2.6%	3.17 (0.32, 31.952)	0.615
Aching pain (n, %)	0, 0%	2, 5.3%	0.95 (0.88, 1.02)	0.493
Pricking pain (n, %)	6, 15.8%	10, 26.3%	0.53 (0.17, 1.63)	0.260
Stabbing pain (n, %)	5, 13.2%	2, 5.3%	2.73 (0.50, 15.03)	0.430
Sleep disorder (n, %)	0, 0%	6, 15.8%	0.84 (0.73, 0.97)	0.025*

*PVB* Paravertebral block, *D* Difference, *CI* Confidential interval, *NRS* Numerical rating scale

^*^Significant statistical difference

At postoperative three months, paravertebral block group experienced less hypoesthesia (OR 0.28, 95% CI 0.11 to 0.75, *P* = 0.009), numbness (OR 0.26, 95% CI 0.07 to 0.88, *P* = 0.024) and sleep disorder (OR 0.84, 95% CI 0.73 to 0.97, *P* = 0.025) than control group. Other recovery data including the rate, severity and characteristics of pain were similar between the two groups (all *P* > 0.05).

## Discussion

The study results showed that perioperative intermittent bolus paravertebral block could provide good anesthetic- and opioid-sparing effects, and enhance postoperative recovery both in-hospital and after discharge in patients undergoing open hepatectomy for hepatic tumor. Intermittent bolus paravertebral block reduced postoperative intravenous opioid consumptions, provided good postoperative analgesia, and reduced rates of hypoesthesia and numbness three months after discharge.

Intermittent bolus paravertebral block reduces postoperative 48 h intravenous morphine consumption in patients undergoing open hepatectomy for hepatic tumor. A previous study using continuous infusion modality showed that opioid consumption was reduced by 21% at postoperative 24 h [9]. Several studies suggested that analgesics delivered via intermittent bolus modality provided comparable or even superior pain relief to analgesics delivered via continuous infusion modality [15–17]. Our study used an intermittent bolus infusion modality, and the results showed that opioid consumption was reduced by 50% at postoperative 24 h. Potential explanations were considered including a wide sensory block range and good maintenance of the block range. The equivalent NRS in later postoperative follow-up period (12/24 to 48 h) implied that the pain was less severe on postoperative day two than one, thus with a higher intravenous opioid consumption, the control group achieved a similar analgesic effect to the PVB group. However, simple PCIA failed to achieve an analgesic effect equivalent to PCIA plus PVB on postoperative day one, thus both the pain NRS and opioid consumption were higher in the control than PVB group on postoperative day one.

Paravertebral block also had an impact on intraoperative hemodynamics and anesthetic management. A previous study on mastectomy and thoracoscopic surgeries showed that paravertebral block reduced intraoperative sevoflurane and opioid consumption, but changes in heart rate and blood pressure were not reported [18, 19]. Our study on patients undergoing hepatectomy showed that the mean arterial pressure of paravertebral block group was lower than that of control group, but similar to its baseline level. As for intraoperative management, although no difference in fentanyl consumption was detected between the two groups, paravertebral block group had lower rest and active pain scores than control group at postoperative 0-h. These results showed that paravertebral block provided better intraoperative analgesia with acceptable hemodynamic fluctuation.

To the best of our knowledge, the current literature does not include any study reporting the effects of paravertebral block on persistent post-surgical pain and recovery after discharge in hepatectomy. The reported effects of paravertebral block on persistent post-surgical pain in other types of surgeries were controversial [11, 20]. While one study on patients undergoing mastectomy suggested that paravertebral block could not reduce the incidence of chronic pain at postoperative three and six months, but reduced the pain score and improved the overall health-related quality of life [21], the other study suggested that preemptive paravertebral block reduced the prevalence of persistent post-surgical pain one year after mastectomy, regardless of whether axillary dissection was performed [22]. A study on thoracotomy suggested that paravertebral block could not reduce chronic postoperative pain [23]. Our study found that paravertebral block did not affect the incidence, severity and characteristics of pain, but reduced the incidence of hypoesthesia and numbness three months after hepatectomy. Possible explanations might be reduced central sensitization due to nerve block, which should be applied as early as possible [21]. Further studies with larger sample sizes and longer follow-up time are required to fully illustrate this issue.

This study has several limitations. First, the early postoperative paravertebral analgesia effect was a dual effect of the initial loading dose and subsequent intermittent bolus dose, so it is unknown if a single injection could achieve a non-inferior analgesic effect. Second, to enable blinding, we did not assess the sensory blockade level after paravertebral block, hence the exact block range was unclear. However, considering that all the blocks were performed by an experienced anesthesiologist under ultrasound guidance, the chances of complete failure were low. Third, since major hepatectomy is associated with a decrease in ropivacaine clearance by > 50% after regional block (transverse abdominal plane block) [24], further studies are required to monitor serum ropivacaine level after paravertebral block. Fourth, we did not exclude patients with preoperative neuropathy at the surgical site, which might violate interpretation of the study results. Fortunately, the baseline past medical history reported no patients with neuropathy history. Also, there might be patients with mild to moderate sleep issues that they felt no need to report as a past medical history during baseline data collection, but they might report it during postoperative three-month follow up when sleep disorder was specifically asked. Fifth, intravenous anesthesia might be more suitable for such a study on pain, to rule out potential influencing analgesic factors of inhalational anesthetics. Sixth, this study was conducted on Asian patients undergoing hepatectomy with a J-shaped incision, the results may not be applied to western patients, hepatectomy with other types of incision or other types of surgeries. Further studies are required to investigate these issues.

## Conclusions

In conclusion, intermittent bolus paravertebral block provided good anesthetic- and opioid-sparing effects, and enhanced recovery both in hospital and after discharge in patients undergoing hepatectomy for hepatic tumor.

## Data Availability

The datasets used and/or analyzed during the current study are available from the corresponding author upon reasonable request.

## Abbreviations

PVB: Paravertebral block
NRS: Numerical rating scale
ICU: Intensive care unit
BMI: Body mass index
ASA: American Society of Anesthesiologists
ALT: Alanine aminotransferase
PT: Prothrombin time
APTT: Activated prothrombin time
